The article "Diagnosis and Treatment Modalities for Osteomyelitis" was retracted in 2024. Reason: plagiarized images.

# Diagnosis and Treatment Modalities for Osteomyelitis

**DOI:** 10.7759/cureus.30713

**Published:** 2022-10-26

**Authors:** Yash Jha, Kirti Chaudhary

**Affiliations:** 1 Orthopedics, Jawaharlal Nehru Medical College, Datta Meghe Institute of Medical Sciences, Wardha, IND; 2 Anatomy, Jawaharlal Nehru Medical College, Datta Meghe Institute of Medical Sciences, Wardha, IND

**Keywords:** treatment of osteomylitis, diagnosis of osteomylitis, chronic osteomylitis, vertebral osteomylitis, osteomylitis

## Abstract

Osteomyelitis is an infection-related inflammatory disease of the bones. Imaging and laboratory results are typically used to support a clinical diagnosis of osteomyelitis. Microbial cultures and bone biopsies provide conclusive diagnoses. The first imaging procedure that needs to be done is radiography, but its sensitivity is low in the early stages of the disease. The sensitivity of magnetic resonance imaging, both with and without contrast material, is higher for detecting areas of bone necrosis in advanced stages. Patients can be categorised for surgical treatment using a staging system based on major and minor risk factors. The main course of treatment should be antibiotics, which should be chosen depending on the findings of the culture and the characteristics of each patient. Bony debridement surgery is frequently required, and in high-risk patients or those with severe illness, additional surgical intervention can be necessary. Better outcomes are being attained in the treatment of this illness thanks to advancements in surgical treatment, antibiotic therapy, and the current resources for precise diagnosis and tailored responses to each kind of osteomyelitis.

The classification systems that are most frequently employed, as well as the general epidemiological ideas, are presented together with the discussion of acute and chronic osteomyelitis. The key recommendations for diagnosing infections clinically, in the laboratory, and through imaging are covered, along with the recommendations for surgical and antibiotic procedures, and the function of hyperbaric oxygen as adjuvant therapy. We evaluate the osteomyelitis-related articles, summarise the most recent developments in diagnostic procedures and therapeutic regimens, evaluate the benefits and drawbacks of various diagnostic modalities and therapeutic approaches, and suggest areas of focus to help current diagnostic and therapeutic approaches.

## Introduction and background

Infection and inflammation of the long bone or the bone marrow are called osteomyelitis. It may occur if a bacterial or fungal infection gets into the bone tissue through the bloodstream after an operation or other trauma. An open wound is the source of development in 80% of cases. Although the sickness can strike anyone, children are more likely to contract it [1]. One of the most prevalent bone infection disorders, post-traumatic osteomyelitis is a sequel to open fractures brought on by a traffic accident, a machine injury, or both. It is also the primary symptom of the postoperative infection of open fractures. Osteomyelitis is easily caused by bacteria that enter the bone tissue after damage and multiply quickly in huge numbers [2]. With an incidence of 21.8 per 100,000 people/year in the United States, osteomyelitis is one of the most difficult conditions for both doctors and patients [3]. The overall incidence of native vertebral osteomyelitis (NVO) was 2.4 per 100 000 in a research from France. Incidence rises with ageing, peaking at 6.5 per 100,000 in patients 50 to 70 years old [4]. Only 10% of all occurrences of osteomyelitis and 1%-6% of all hand infections involve osteomyelitis of the hand [5].

## Review

Classification

An ideal classification of osteomyelitis would cover all potential etiologies and dimensions of temporal evolution, taking into account the various factors that affect its pathophysiology [6]. As osteomyelitis is a heterogeneous disease; there are more than 12 possible categories due to the wide range of patient populations and a number of other criteria that are important for determining the best course of treatment. Two classifications are frequently used despite the fact that none of them are universally acknowledged. This is because they offer details on the nature and causation of the disease while also taking into account the patient's physiological state, two factors that are crucial in osteomyelitis. Osteomyelitis treatment is largely dictated by whether it is considered "acute" or "chronic" in the clinical environment. The degree of tissue harm is typically directly connected with the illness stage, despite the fact that there is sometimes great difficulty in this classification. The Waldvogel system and the Cierny-Mader system are the two most frequently mentioned detailed classification systems for illness that have been published in the literature [7]. In general, the Cierny and Mader classification is advised due to its well-defined surgical treatment ideas, however, the Waldvogel classification is suggested due to its wider clinical relevance [6].

Waldvogel Classification

According to the Waldvogel classification system, an infection is classified as either acute or chronic depending on how persistent it is. The classification is then made based on the source of the infection. According to Waldvogel et al., this definition not only revealed evidence of variations in clinical presentation but also increased the likelihood that a condition would be cured [7].

Cierny-Mader Classification

The four main components of the Cierny-Mader categorization system are the state of the host, the functional impairment brought on by the illness, the place of involvement, and the degree of bony necrosis. It does not believe that a distinction between acute and chronic infections is necessary. There are 12 clinical staging systems for adult osteomyelitis as a result of this classification system. The osteomyelitis treatment, which entails debridement techniques, managing dead space, and giving antibiotics, is adapted from this staging approach. According to Cierny et al., comparing novel treatment protocols and the efficacy of new therapy modalities is made possible by considering these four crucial parameters [7].

Types

The optimal course of action is determined by how severe the osteomyelitis is, which can be either acute or chronic. Acute osteomyelitis patients often show without bone deterioration days to weeks after the initial infection, with symptoms including pain, fever, and edoema at the afflicted site. After several months to years of ongoing infection, chronic osteomyelitis can manifest as necrotic bone and fistulous passages connecting the skin to the bone.

Hematogenous or nonhematogenous infection mechanisms are used to further categorise osteomyelitis. Hematogenous osteomyelitis is a disorder when germs enter the bone as a result of a bloodstream infection. Immunocompromised people, children, and older people are more likely to develop this condition. Vertebral osteomyelitis is the most prevalent type of hematogenous osteomyelitis; patients frequently have back or neck discomfort, muscle aches, and occasionally fever. The long, pelvic, and sternoclavicular bones are other bones where hematogenous osteomyelitis can develop. Prepubescent children who suffer from hematogenous osteomyelitis often experience it in the metaphysis of long bones close to growth plates, with the tibia and femur being particularly susceptible. Nonhematogenous osteomyelitis is caused by direct inoculation during surgery, after trauma, or as a result of spreading infections in nearby soft tissues and joints [1].

Diagnosis

The case below was taken through different imaging techniques thereby showing an ideal case of chronic osteomyelitis (Figure 1).

**Figure 1:** Chronic osteomyelitis of the tibia in a 16-year-old female Images taken through (A) conventional radiography (B) CT scan (C) MRI (D) MRI. Image taken by Yash Jha.

Orthopaedic doctors find it challenging to diagnose and treat this illness. Immune techniques in combination with imaging techniques (such as CT and MRI) have greatly increased the diagnostic precision and capability of early diagnosis in recent years [2].

These steps can be followed for diagnosis of osteomyelitis:

1. Conduct a thorough neurological assessment.

2. Perform a laboratory assessment, including two sets of blood cultures, complete blood count (CBC), erythrocyte sedimentation rate (ESR), C-reactive protein (CRP), basic metabolic panel, urinalysis, and urine culture.

3. If the patient has abnormal neurological findings, get urgent bone imaging; if normal, get it within six hours. Options for imaging include:

i) The best imaging investigation is an MRI of the whole bone, with and without contrast. If contrast might slow down imaging, leave it out.

(ii) Get an immediate CT myelogram if an MRI is not an option (the reason, for example, could be due to a huge body mass, or an implanted device, or a metallic foreign object present in the body). 

iii) Perform a CT with IV contrast if a CT myelogram is not an option.

Note: Due to their poor spatial resolution and specificity, scintigraphy (Technetium-99 bone scans and Gallium-67 scans) and metabolic imaging (FDG CT/PET) are not regarded as major imaging options. Diagnostic lags are common; reports range from 11 to 59 days from symptom start to diagnosis.

4. Get a biopsy. If the blood culture is negative and imaging indicates osteomyelitis, then radiology should perform an urgent or emergency biopsy under the supervision of imaging [8].

Figures 2-7 given below show the affected areas due to osteomyelitis.

**Figure 2:** Staphylococcus aureus osteomyelitis in a 20-year-old man. Images taken through (A) conventional radiograph (B) MRI coronal T1w (C) axial T2w fat-saturated (D) show a permeative lesion of the left femoral shaft; (E) CT scan.

**Figure 3:** X-ray of leg showing osteomyelitis in the fibula Image taken by Yash Jha.

**Figure 4:** X-ray of leg showing osteomyelitis in the tibia Image taken by Yash Jha.

**Figure 5:** MRI of leg showing osteomyelitis in the right tibia Image taken by Yash Jha.

**Figure 6:** MRI of leg showing osteomyelitis in the tibia Image taken by Yash Jha.

**Figure 7:** CT of leg showing osteomyelitis in the lower tibia Image taken by Yash Jha.

Garre's osteomyelitis which frequently affects the unilateral mandibular body, develops in young individuals mostly as a result of odontogenic infections. The mandible's premolar and molar areas are most frequently affected. Bone hyperplasia and destruction are imaging findings in Garre's osteomyelitis of the jaws, and some of these findings resemble the X-ray presentations of malignant tumours [9]. Typically, the metaphyseal region of long bones is where osteomyelitis originates (or long bone equivalent areas, such as the calcaneal apophysis or inferior pubic ramus). Osteomyelitis and septic arthritis occur together at a 33% prevalence [10]. The development of osteomyelitis is also influenced by host defences. Systemic illnesses like diabetes, autoimmune conditions, cancer, malnutrition, and AIDS have all been linked to osteomyelitis [11]. When bone pain and inflammation are not appropriately treated, children may have impaired physical function and poor attendance at school. Skeletal injury that is permanent can result from delayed diagnosis. Most people are still unsure of the exact aetiology of the illness, however, immune dysregulation is thought to have a role in the inflammation of bones, as well as other tissues occasionally, like the skin, joints, and intestines [12]. Early signs of diabetic foot osteomyelitis are nonspecific, and any diabetic patient who complains of foot discomfort, tenderness, redness, warmth, or induration should be evaluated for infection, particularly if an open lesion is present. By spreading continuously from the soft tissue, bone infection is possible [13].

Treatment

The main course of treatment should be antibiotics, which should be chosen depending on the findings of the culture and the characteristics of each patient [1]. Orthopedic physicians and patients have new treatment options with cutting-edge reconstruction and repair techniques like Ilizarov and Orthofix LRS. Surgery used to try to remove infected and necrotic bone worsens the patient's condition [2]. As a result of new biomaterials entering the market, such as bioactive glass S53P4 (BonAlive®, Bonalive Biomaterials Ltd., Turku, Finland) and CeramentTM G (Bonesupport, Lund, Sweden), osteomyelitis therapy is gradually moving from a two-stage to a one-stage approach in the Western world [14]. If an imaging examination reveals osteomyelitis, then start antibiotics right away. If the patient has unstable hemodynamics, then hold off on antibiotics until after the biopsy of the patient is hemodynamically stable, unless the blood cultures are positive. Consider consulting a neurosurgeon and every four hours, conduct a neurological examination. If the patient's hemodynamics are stable and no encouraging microbiological or imaging results are found, then keep other diagnoses in mind and repeat imaging in 1-3 weeks if discomfort is persistent.

Medical treatment entails correcting any host inadequacies, choosing an initial antibiotic, and modifying that antibiotic based on culture results. Effective oral drugs and local therapy using antibiotics combined with polymethylmethacrylate have both been added to the repertoire of antibiotic delivery methods [15]. The selection of antibiotics is complicated by the rise of methicillin-resistant Staphylococcus aureus (S. aureus) osteomyelitis. In chronic situations, surgical debridement is typically required. Even after surgical intervention and prolonged antibiotic medication, the recurrence rate is still significant. A four-week course of antibiotics is often effective in treating acute hematogenous osteomyelitis in children [16]. Bacteremic bone seeding causes acute hematogenous osteomyelitis. Because the metaphyseal (developing) portions of the long bones are extremely vascular and sensitive to even slight damage, children are most frequently impacted. Acute hematogenous osteomyelitis affects children under the age of five in more than half of cases [16]. Treatment with antibiotics can be given intravenously or orally [17]. The best type, method of administration, and length of antibiotic therapy are still debatable, and the rise of multi-drug resistance pathogens presents significant therapeutic difficulties. The fate of patients is significantly influenced by the determination of the underlying cause and subsequent targeted antibiotic therapy [18].

To get high doses of the medication into the blood, antibiotics are typically administered initially by IV. In the future, antibiotic pills might be taken. Antibiotics are typically required for four weeks for children. Antibiotics must be taken for six to eight weeks by adults [19]. The therapy of osteomyelitis was well-reviewed by Drs. Hatzenbuehler and Pulling. One crucial tool, which is useful for chronic diseases was left out. In patients with persistent refractory osteomyelitis, hyperbaric oxygen treatment (HBOT) is linked to remission rates of 81% to 85% at two to three years. It entails putting the patient in a single or multiple-person chamber where he or she is exposed to higher atmospheric pressure while breathing only 100% oxygen. A typical therapy course consists of five 90-minute sessions over the course of 20 to 60 sessions. Enhanced leukocyte oxidative killing, osteogenesis, angiogenesis, and synergistic antibiotic activity are the mechanisms of action. Treatment complications are rare, and pneumothorax and prior bleomycin therapy are the only absolute contraindications. Local hyperbaric resources should be known to family doctors, who should consider using this treatment for the right patients [20]. Before attempting more extensive surgical treatments, culture-directed antibiotics and HBO2 therapy offer a reasonable chance of curing osteomyelitis. In general, HBO2 therapy is administered once per day, five to seven days a week, for 90 to 120 minutes, at 2.0 to 3.0 atmospheres absolute (ATA) pressure. The current antibiotic and HBO2 therapy regimen should be continued in cases where rapid clinical improvement is observed for a period of four to six weeks; 20-40 HBO2 treatments are often needed to produce long-lasting therapeutic benefits [21].

Hospitalization rates range from 1.34 to 1.66 per 100,000 kids annually, with the annual incidence estimated to be between 2 and 13 per 100,000 kids. With an incidence of 43 to 80 cases per 100,000 kids, paediatric osteomyelitis represents a substantially greater healthcare burden from a global health perspective. Lower extremities and long bones, particularly the femur (23% to 29%), tibia (19% to 26%), humerus (5% to 13%), pelvis (3% to 14%), and calcaneus (4% to 11%), are the most often affected locations. Children with osteomyelitis are usually male and their age is below five years [22]. Every case of osteomyelitis results in a significant socioeconomic burden as well as a potential existential threat to the affected patient. According to some studies, the cost of treatment could reach €500,000 per case [23]. Revascularization may be required in some patients because the treatment of diabetic foot osteomyelitis is frequently worsened by ischemia of the affected limb as a result of peripheral vascular dysfunction [24].

For the best results, antibiotics must be taken as soon as possible, before there is significant bone loss or necrosis. This requires parenteral administration of the medication for at least four weeks, but ideally six [25]. The rise of invasive community-acquired methicillin-resistant S. aureus infections is modifying the clinical presentation and treatment of osteomyelitis in children and adolescents. Treatment with antibiotics should target S. aureus, including methicillin-resistant forms acquired in the community [26]. In addition to antibiotic therapy, surgical debridement is required for the treatment of chronic osteomyelitis since it is characterised by avascular necrosis of the bone and the development of sequestrum (dead bone) [25].

Clinical characteristics that raise suspicion for osteomyelitis are limb weakness, dysesthesias, radicular pain, gait disturbance, and bowel or bladder dysfunction [1]. The factors which increase the risk of osteomyelitis are provided in Table 1.

**Table 1:** Factors which increase the risk of osteomyelitis

	Factors which increase the risk of osteomyelitis
1	cardiovascular disease
2	Rheumatoid arthritis
3	History of trauma or fracture
4	HIV or AIDS
5	Malignancy
6	Smoking or alcohol use
7	diabetic foot ulcers
8	Cirrhosis or chronic kidney disease
9	Peripheral vascular disease and poorly healing wounds (e.g., decubitus ulcers)
10	Any risk factor for bacteremia (eg, IV drug use or an indwelling vascular device)
11	Diabetes mellitus (the most common risk factor) [27].

Chronic nonbacterial osteomyelitis (CNO)

Children and teenagers are most frequently affected by chronic nonbacterial osteomyelitis (CNO), an inflammatory bone condition. A severe variant of CNO known as chronic recurrent multifocal osteomyelitis (CRMO) is characterised by symmetrical inflammatory bone lesions and a waxing and waning pattern [28]. Clinical symptoms can include pathological fractures, localised bone pain, localised swelling, seldom cutaneous redness and heat, and related skin manifestations (such as palmoplantar pustulosis, psoriasis, and acne) [29]. There are no drugs approved for use in CNO at the moment. Most patients respond to nonsteroidal anti-inflammatory medications (NSAIDs) in some way, but other patients need more severe therapy, which may involve corticosteroids, cytokine-blocking medications, or bisphosphonates. NSAIDs are frequently utilised as first-line treatments in patients whose vertebral columns are uninvolved. In a small percentage of CNO/CRMO patients, NSAIDs effectively decrease bone inflammation and offer comparatively rapid clinical relief. However, within two years of starting treatment, more than 50% of CNO/CRMO patients experience flare-ups when using NSAIDs. NSAIDs to variable degrees, inhibit cyclooxygenase (COX) enzymes and decrease inflammasome assembly. In limited cohorts of CNO/CRMO patients, it has been reported that corticosteroids, DMARDs (sulfasalazine and methotrexate), biologic therapies (anti-TNF medicines), and bisphosphonates are efficacious [28].

Optimal cutoff values for ESR and CRP in patients with diabetes-related foot infections to diagnose osteomyelitis

Based on the findings of the resuscitation outcomes consortium (ROC) analysis, the ideal cutoff values for predicting osteomyelitis were determined to be an ESR of 60 mm/h and a CRP level of 7.9 mg/dL. While the CRP threshold of 7.9 mg/dL had a sensitivity of 49% and specificity of 80% for osteomyelitis, the ESR threshold of 60 mm/h showed a sensitivity of 74% confidence interval, and 56% for osteomyelitis. Osteomyelitis is unlikely if the ESR is less than 30 mm/h. However, there is a significant risk of osteomyelitis if the ESR is greater than 60 mm/h and the CRP level is greater than 7.9 mg/dL, then treatment of suspected osteomyelitis should be strongly considered.

While CRP can help patients with high ESR readings identify osteomyelitis from soft-tissue infection, ESR is still preferable for initially ruling out osteomyelitis. ESR and CRP prognostic usefulness requires further prospective research, and a more complete diagnostic algorithm should be created to incorporate additional diagnostic tests such as imaging and probe-to-bone [30].

## Conclusions

We provide more clarity about osteomyelitis which is an inflammation of the long bone and bone marrow. Although it is a rare disease, its cases are increasing rapidly. The Waldvogel system and the Cierny-Mader system are the two most frequently mentioned classifications even though none of them are universally acknowledged. The optimal course of action is determined by how severe osteomyelitis is, which can be either acute or chronic. Hematogenous or nonhematogenous infection mechanisms are used to further categorise osteomyelitis. Doctors find it challenging to diagnose and treat this illness. We have mentioned some of the diseases that make patients prone to osteomyelitis. Immune techniques in combination with imaging techniques (CT and MRI) have greatly increased the diagnostic precision and capability of early diagnosis in recent years. We have explained the diagnosis process step-by-step with the preference order which is required to be followed. We have also explained refractory osteomyelitis, HBOT, and other treatments which are required to be followed depending on the condition of the patient.
